# Pharmacovigilance with Transformers: A Framework to Detect Adverse Drug Reactions Using BERT Fine-Tuned with FARM

**DOI:** 10.1155/2021/5589829

**Published:** 2021-08-13

**Authors:** Sajid Hussain, Hammad Afzal, Ramsha Saeed, Naima Iltaf, Mir Yasir Umair

**Affiliations:** National University of Sciences and Technology (NUST), Islamabad, Pakistan

## Abstract

Adverse drug reactions (ADRs) are the undesirable effects associated with the use of a drug due to some pharmacological action of the drug. During the last few years, social media has become a popular platform where people discuss their health problems and, therefore, has become a popular source to share information related to ADR in the natural language. This paper presents an end-to-end system for modelling ADR detection from the given text by fine-tuning BERT with a highly modular Framework for Adapting Representation Models (FARM). BERT overcame the predominant neural networks bringing remarkable performance gains. However, training BERT is a computationally expensive task which limits its usage for production environments and makes it difficult to determine the most important hyperparameters for the downstream task. Furthermore, developing an end-to-end ADR extraction system comprising two downstream tasks, i.e., text classification for filtering text containing ADRs and extracting ADR mentions from the classified text, is also challenging. The framework used in this work, FARM-BERT, provides support for multitask learning by combining multiple prediction heads which makes training of the end-to-end systems easier and computationally faster. In the proposed model, one prediction head is used for text classification and the other is used for ADR sequence labeling. Experiments are performed on Twitter, PubMed, TwiMed-Twitter, and TwiMed-PubMed datasets. The proposed model is compared with the baseline models and state-of-the-art techniques, and it is shown that it yields better results for the given task with the *F*-scores of 89.6%, 97.6%, 84.9%, and 95.9% on Twitter, PubMed, TwiMed-Twitter, and TwiMed-PubMed datasets, respectively. Moreover, training time and testing time of the proposed model are compared with BERT's, and it is shown that the proposed model is computationally faster than BERT.

## 1. Introduction

Adverse drug reactions (ADRs) according to the definition of the World Health Organization (WHO) are a response to noxious medication which occurs as a result of normal doses used in man for diagnosing or curing a disease [1]. ADRs greatly affect quality of life and in worse cases can be a cause of death. A study showed that 3.5% of the patients were hospitalized because of ADRs [2]. It has been estimated that ADRs were responsible for approximately 197,000 deaths annually in Europe [3]. The safety of a drug is monitored by the Food and Drug Administration (FDA) after its release. *Pharmacovigilance, also known as drug safety, is the pharmacological science relating to the collection, detection, assessment, monitoring, and prevention of adverse effects with pharmaceutical products* [4]. These surveillance activities, however, are largely reliant on a passive spontaneous reporting database known as Adverse Event Reporting System (AERS) [5]. Delayed and underreported events can make these systems inefficient.

To address the limitations of passive surveillance, active pharmacovigilance techniques used for labeling ADRs analyze frequently updated sources of data. Data from social media particularly Twitter because of its public nature and vast reach can be used as a source of carrying out postmarket drug surveillance. Studies have observed significant correlations between ADRs reported in AERS and those mentioned in Twitter [6]. Several studies have been conducted on Twitter data [7, 8]; however, limitations arise due to the informal language of social media. As compared to Twitter, a very formal description is found in biomedical text. Hence, some studies use biomedical text collected from PubMed abstracts for ADR extractions [9, 10], while some utilize data from both social media and biomedical text [11, 12]. In this work, we also use datasets from both sources, i.e., Twitter and PubMed.

ADR extraction has been performed using conventional machine learning models such as Support Vector Machine (SVM) [13], Random Forest (RF) [14], and Conditional Random Field (CRF) [15]. These models depend upon manual feature engineering. The most common features utilized by these models include *n*-grams, negated contexts, semantic types from the Unified Medical Language System (UMLS), Part of Speech (POS) tags, drug names, lexicon-based features, and word embeddings [16]. Numerous studies utilize deep learning techniques such as Bidirectional Long Short-Term Memory (BLSTM) [12], Convolutional Neural Network (CNN) [17], and attention-based deep neural networks [11]. Most recent studies have employed Bidirectional Encoder Representations from Transformers (BERT) and its different variants which significantly improved the performance of ADR detection [8, 18]. However, despite an increase in the accuracies, BERT is computationally expensive and has a slower speed at inference time which limits its usability. A study observed that the BERT_base_ model took about 1.7 seconds to classify a single piece of text on a Google Pixel 3 smartphone [19]. For industrial purposes, billions of requests need to be processed per second in the tasks like text classification. This makes the usage of BERT impractical for production environments. Moreover, it also requires a large amount of time for training which limits the tuning of hyperparameters. Hence, determining the most contributing hyperparameters becomes challenging. Furthermore, ADR extraction from social media data firstly requires text classification to remove noise and filter text with ADR mentions. Text classification is then followed by the task of ADR sequence labeling. Hence, a framework with the support of multitask learning is needed for end-to-end modelling of the problem.

In this work, we use BERT fine-tuned via a novel framework FARM (https://farm.deepset.ai/) to detect ADRs on Twitter and PubMed datasets. FARM supports parallelized processing which makes the model computationally faster and hence practical for industrial purposes. The hyperparameters used in the standard BERT model are modified with FARM-BERT such that they best fit the learning task. FARM has a modular design for language models and prediction heads which makes transfer learning simpler. FARM is an adaptive model that provides support for combining multiple prediction heads on top of the language model. We present an end-to-end solution for ADR extraction by using two prediction heads with BERT, one for classifying text with ADR mentions and the other for labeling ADR sequences in the classified text. In short, primary contributions of this work are listed below:

- A FARM-BERT based on a highly modular design is utilized to detect ADRs
- A framework with the support of multitask learning using two prediction heads is proposed for end-to-end modelling of the problem
- A computationally fast solution is proposed to detect ADRs which support parallelized processing and learn faster on big datasets as compared to the traditional BERT
- FARM-BERT is fine-tuned with different sets of hyperparameters as compared to the standard BERT
- Comparison of results shows that BERT fine-tuned using FARM outperforms state-of-the-art techniques used for extracting ADRs

The rest of the paper is structured as follows: Section 2 presents the literature review, Section 3 proposes a framework for end-to-end detection of ADRs, and Section 4 discusses experiments and results while Section 5 draws the conclusion.

## 2. Literature Review

There has been a considerable amount of work for detecting ADRs from biomedical text automatically using machine learning approaches. Earlier works utilize traditional machine learning approaches with manual feature engineering. Liu and Chen [13] passed bag of words, bigrams, and Part of Speech (POS) tags as features to SVM where the bag of words produced the best results. The bag of words approach is based on the occurrences of words in a corpus. It ignores the semantics and syntax of the text. Hence, this approach is not a reliable approach leading to false classifications. Alimova and Tutubalina [20] fed SVM and Logistic Regression (LR) with features including lexicon-based features, sentiment features, semantic features, and word embeddings. Since lexicon is based on a particular list of drugs, lexicon-based features do not play a significant role in ADR identification. Sentiment and word embedding features have been found to be the most effective. Sarker and Gonzalez [21] used SVM fed with topic model features in combination with other features such as *n*-grams, sentiword scores, lexicon features, synset expansion features, and UMLS semantic types. Bian et al. [22] also used semantic features based on UMLS in combination with other textual features. In the shared task Social Media Mining for Healthcare (SMM4H) 2017, the best performing system employed SVM fed with different domain-specific, surface-form, and sentiment features [23]. Aramaki et al. [24] used SVM and CRF for extracting adverse drug effects using lexicon-based features, POS tags, word chain, etc. CRF has also been used in [15] which utilized contextual features, word embedding features, and dictionaries. Another approach [14] uses the RF model fed with *n*-gram features, negation, sentiment, etc. Traditional approaches rely upon manual feature engineering which needs considerable effort and time.

Recent approaches for ADR detection employ deep neural networks. CNN initialized with Pyysalo's word embeddings [25] has been used in [17] to detect ADRs. Chowdhury et al. [26] proposed the Convolutional Recurrent Neural Network (CRNN) for ADR detection. In [12], the BLSTM network was used with word embeddings as input features. In [26], a multitask encoder-decoder framework has been proposed that provides end-to-end solution by modelling three ADR detection tasks, i.e., classification of ADRs, ADR labeling, and indication labeling. To tackle the problem of limited labeled data for ADR, Gupta et al. [27] proposed a semisupervised approach based on cotraining which can augment the labeled data with a large amount of unlabeled data. A semisupervised model was also proposed in [28]. For the unsupervised learning stage, the drug name was predicted on the basis of its context in the given tweet using the BLSTM model. The BLSTM model initialed with word2vec-based word embeddings was trained in the supervised learning stage to predict the sequence labels in tweets. Zhang and Geng [29] presented a weakly supervised CNN-LSTM model to identify ADRs. Weakly labeled data was employed to pretrain the model. The model parameters were further fine-tuned on the labeled dataset. Some models combine deep neural networks with traditional models such as BLSTM-CRF for sequence labeling [30]. They exploit both word embedding-based features and other natural language processing features such as spelling features, *n*-gram features, and POS features. Another BLSTM-CRF model uses character embeddings in addition to word embeddings [31]. In [32, 33], combination of CNN, LSTM, and CRF has been proposed where word embeddings are augmented using character level CNN.

Neural network models, when processing long texts, suffer from the problem of vanishing gradient. The problem can be dealt with using an attention mechanism. In the attention mechanism, the decoder retrieves selective information from the most relevant parts of the source sentence instead of using all the information encoded into a fixed-sized vector [34]. Ramamoorthy and Murugan [9] proposed a self-attention-based BLSTM model for facilitating intrasequence interaction in the given text sequence. Ding et al. [11] proposed the embedding level attention mechanism in the Bidirectional Gated Recurrent Unit (BGRU) to allow the model to learn the most important features. The recent meeting of SMM4H held in 2019 showed further improvements in neural network techniques used for ADR detection [35]. Convolutional and recurrent neural architectures fed with word2vec or glove embeddings being the most popular architectures for tackling the task in 2018 were overtaken in 2019 by neural networks that used word embeddings pretrained with BERT [36]. The approach of the winning team was based on retraining BERT on a large unlabeled tweet dataset collected from Twitter using a list of drug names [37]. In [8], domain-specific preprocessing and an ensemble of different BERT implementations, i.e., general BERT_LARGE_, domain-specific BioBERT [38], and domain-specific ClinicalBERT [39], have also been shown to be effective for ADR classification on social media. Li et al. [18] integrated BERT with CNN and utilized emotional information to distinguish between ADR and non-ADR tweets. Aroyehun and Gelbukh [7] used LSTM fed with a combination of three types of embeddings, i.e., character embeddings, glove embeddings, and BERT embeddings, to detect ADR reportage in tweets. Informal expression in social media text makes ADR detection a challenging task. To mitigate the effect of such informality, Zhang et al. [40] proposed an adversarial transfer network with bilinear attention which transfers auxiliary information from the PubMed dataset to social media datasets. Kang et al. [41] proposed entity recognition of ADRs in Chinese text by constructing a model comprising self-attention, adversarial transfer learning, RNN, BLSTM, and CRF.

ADR mentions are mostly overlapping and discontinuous which makes ADR extraction a difficult task. To overcome this issue, El-allaly et al. [42] proposed a deep neural network named as DeepCADRME which tackles ADR extraction as an *N*-level tagging sequence problem and transfers knowledge between the levels. The sequences are fed to the *N*-level model on the basis of contextual embeddings in which output of the current level's pretrained model is used to create a new contextualized representation for the following level.

## 3. Proposed Methodology

We use BERT implemented via a novel framework FARM to detect ADRs. This section briefly discusses the architecture of BERT followed by a brief description of the pretrained BERT used in our study. We then describe the fine-tuning of BERT with FARM.  Figure 1 presents the overall architecture of the proposed system.

### 3.1. BERT

Training BERT involves two phases, i.e., pretraining and fine-tuning. In the first phase, i.e., pretraining, unlabeled data is used to train the model over different tasks. In fine-tuning, the pretrained parameters are fine-tuned on the labeled dataset to model a downstream task. The architecture of BERT is based on bidirectional transformers in multiple layers [43]. In this work, we use BERT_base_ which consists of 12 layers denoted as *L*, 768 hidden units denoted as *H*, and 12 self-attention heads denoted as *A*.

### 3.2. Input Representation

BERT generates contextualized embeddings. Many models have widely been used to convert words into embeddings such as word2vec, fasttext, and glove. However, these models generate embeddings of a word without considering its context. In natural language, meanings of a similar word may vary in different contexts. Context-dependent representation is not captured by these models resulting in similar vector representations of a word having different meanings in different contexts. As opposed to the previous models, BERT generates contextualized embeddings.

BERT takes as input a single sentence or a pair of sentences. BERT uses the WordPiece model to tokenize the input sequence. Special tokens are added by the tokenizer at the beginning and end of the input sequence. The first token that marks the beginning of every input sequence is [*CLS*]. Two sentences in the input sequence are divided by a special token [*SEP*]. Besides tokenizing the input sentences into words, individual words, if not found in the vocabulary, are also tokenized into subwords and characters. In this way, BERT generates embeddings out of vocabulary words by generating embeddings of their constituent subwords and characters found in the vocabulary. In addition to producing the token embeddings, BERT generates sentence embeddings by adding embedding to each token in the tokenized text indicating whether the token belongs to the first or the second sentence. It further generates position embeddings indicating the position of a token in the input sequence. Finally, the input representation for a given token can be represented by concatenating its corresponding token embeddings, sentence embeddings, and position embeddings.

Let *t*_*i*_ represent the token embedding of the word *i* and *s*_*i*_ represent its sentence embedding while *p*_*i*_ represents its position embedding, then the embedding of a word *i* denoted as *E*_*i*_ can be represented as follows:

(1) $$\begin{array}{c} E_{i}=ti⊕s_{i}⊕p_{i}, \end{array}$$

where ⊕ represents the concatenation operator.

### 3.3. Pretrained BERT

We use the general purpose BERT model pretrained on BBC news corpus. Pretraining BERT comprises two supervised tasks. In the first task, BERT uses the concept of masking to mask some input tokens randomly and predict the masked tokens, hence learning bidirectional representations. The hidden representations of the masked tokens are passed to the softmax layer. The second task is next sentence prediction, the purpose of which is to understand the relationship between two sentences.

### 3.4. Fine-Tuning BERT with FARM for ADR Detection

Transfer learning represents the idea of adapting learning from one task to another. Knowledge learned by the pretrained BERT model can be used to model any downstream task. We use FARM to fine-tune BERT for detecting ADRs from the given text sequences. FARM provides a framework that makes transfer learning with BERT simpler. It is built using transformers and provides a modular design for the language models and prediction heads. The process is divided into the following two phases.

#### 3.4.1. Data Handling

The modular structure of FARM makes preprocessing quite convenient and customizable as compared to BERT's wordpiece tokenization which follows the conventional HuggingFace approach. Processors are utilized to transform input files into PyTorch datasets. For this purpose, a tokenizer is required by the processor which can be loaded based on the required language model.

#### 3.4.2. Modelling

FARM provides a generalized and flexible approach of transfer learning. The adaptive model of FARM provides a framework for end-to-end transfer learning. It combines the following two components, i.e., language model and the prediction heads.

- *Language Model*. A pretrained language model such as BERT and XLNet converts tokens into vector representations. As mentioned earlier, the pretrained language model used in our case is BERT_base_.
- *Prediction Head*. A prediction head is the layer on top of the language model which is used for modelling the downstream task. The vector representations from the language model are fed to the prediction head which converts them into the predictions of the downstream task.

The pretrained language model is adapted to the downstream task using the prediction heads. The downstream task in our case is ADR extraction. FARM simplifies multitask learning by allowing to switch between multiple prediction heads on top of the language model. Using FARM, any pretrained language model such as BERT and XLNet can be attached to one or more prediction heads such as the NER head and classification head. Two prediction heads are used in the proposed model, one for text classification in which the text samples mentioning ADRs are detected and the other for ADR sequence labeling in which a label is predicted for each token in the given sequence of tokens of the input text.

During training, the model backpropagates the loss through the whole neural network including the language model.

### 3.5. ADR Prediction

Given an input sequence *s*, weight matrix *w*, and bias value *b*, the probability of the given sequence *s* belonging to class *c* is computed by the softmax function as the value of the variable *x*:

(2) $$\begin{array}{c} P\left(x=c\;|\;s;w;b\right)=\text{softmax}\left(w\cdot s+b\right)=\frac{e^{w_{c}\cdot s+b_{c}}}{\sum_{n=1}^{n}w_{n}\cdot s+b_{n}}, \end{array}$$

where *n* denotes the total number of ADR categories.

### 3.6. Optimization

FARM-BERT is optimized using the adam optimizer. The parameter update rule of adam is given as follows:

(3) $$\begin{array}{c} w_{t}=w_{t-1}-\eta \frac{{\hat{m}}_{t}}{\sqrt{{\hat{v}}_{t}}+\varepsilon }, \end{array}$$

where *w* represents weights of the model, *m* represents moving averages, and *η* is the step size.

## 4. Experiments and Results

In this section, we brief the experimental settings of models used for experiments. We also evaluate the models and discuss the results.

### 4.1. Datasets

Experiments are performed on three datasets. The first dataset is the Twitter dataset used in [12] which was created by combining two datasets, i.e., Twitter ADR dataset and Attention Deficit Hyperactivity Disorder (ADHD) dataset. The Twitter ADR dataset was collected using the names of 81 drugs common in the US market [44]. The drugs used in the tweets of this dataset did not represent any specific condition but a wide range of different ADRs. The dataset was supplemented with an additional ADHD dataset which contained the drug names used for treating ADHD. The dataset is divided into 75% train data and 25% test data. Sequence labeling is usually done using the standard I-O-B scheme according to which the tokens are labeled based on their positions either at beginning (B), inside (I), or outside (O) of the given entity. The Twitter data has been labeled by adopting an I-O scheme having 4 categories: I-ADR indicating the given token is a part of an ADR, I-indication indicating the given token is a part of an indication, O-indication indicating the token is outside any indication or ADR, and <PAD> indicating that the token is a padding.

The second dataset comprising biomedical text has been collected from PubMed abstracts [45]. There are 6,821 sentences in the dataset. The dataset is divided into train data, validation data, and test set in the ratio of 8 : 1 : 1. A similar I-O scheme has been used for annotating the PubMed dataset. However, the dataset does not contain any I-indication category leaving behind 3 labels for each token, i.e., I-ADR, O, or <PAD>.  Figure 2 shows the examples of the sentences mentioning ADRs in Twitter and PubMed datasets.

The third dataset is the TwiMed corpus [46]. This dataset further comprises two parts, TwiMed-Twitter and TwiMed-PubMed. Three types of entities are labeled in the corpus, i.e., drugs, symptoms, and diseases. We consider symptoms and diseases as adverse reactions in our experiments. Moreover, there are three types of relations between these entities, i.e., reason-to-use, outcome-negative, and outcome-positive. Outcome-negative indicates that drugs in the given input sequence can be a cause of adverse reactions. We consider the sentence as ADR-positive if the relationship between drugs and adverse reactions was annotated as outcome-negative. Similar considerations have also been made in the experiments conducted by Zhang et al. [47].

Table 1 provides the quantitative details of the datasets used for experiments.

### 4.2. Evaluation Metrics

Precision (*P*), recall (*R*), and *F*-score (*F*) are used to evaluate the performance of the model. We choose these metrics because they have widely been used for evaluating the models in state-of-the-art works.

Precision measures the relevancy of the results. In other words, it describes how many samples predicted to be belonging to a certain class actually belong to that class. It shows how often our model misclassifies other classes as this class:

(4) $$\begin{array}{c} P=\frac{\text{True positives}}{\text{True positives}+\text{false positives}}. \end{array}$$

Recall measures how many actual relevant results have been returned. It calculates how many actual samples belonging to a certain class are correctly predicted by the model giving insight into the misclassification of this class as another class:

(5) $$\begin{array}{c} R=\frac{\text{True positives}}{\text{True positives}+\text{false negatives}}. \end{array}$$

Very often, precision and recall are inversely related to each other. To overcome this imbalance, the *F*-score is used which is the harmonic mean of precision and recall:

(6) $$\begin{array}{c} F=\frac{2\cdot P\cdot R}{P+R}. \end{array}$$

### 4.3. Proposed Model Configuration

The proposed model is implemented in Python programming language using PyTorch library. The learning rate in FARM-BERT is set to 3*e* − 5. The model is fine-tuned using a batch size 8 for 5 epochs.

### 4.4. Comparison with Baseline Models

Experiments are performed with the following conventional and deep learning models on Twitter and PubMed datasets. The results of these models are compared with the proposed model.

- *Support Vector Machine (SVM)*. We use a linear kernel SVM to detect ADR based on word *n*-grams, sentence embeddings, and lexical features, i.e., names of drugs and ADRs.
- *Multilayer Perceptron (MLP)*. We use the MLP classifier fed with word *n*-grams, sentence embeddings, and lexical features, i.e., names of drugs and ADRs. Batch size is set to 16, and adam is used as an optimizer.
- *Convolutional Neural Network (CNN)*. We initialize the embedding layer of CNN with word embeddings. Three filters of heights 3, 4, and 5 are used in the convolutional layer. 1-max pooling is applied over the convolved feature maps to select the most salient features and reduce the output dimension. The resultant features are concatenated and passed to the output layer which detects the presence of ADR in the given input sequences. We use the batch size of 16 and adam as the optimization algorithm.
- *Long Short-Term Memory (LSTM)*. We initialize the embedding layer of LSTM with word embeddings. The sequences returned by this layer are passed to the LSTM layer followed by a dense layer. The final layer is the output layer which uses softmax activation function to detect ADRs. We use batch size of 16 and rmsprop as an optimizer.
- *Bidirectional Encoder Representations from Transformers (BERT)*. BERT is a bidirectional transformer encoder having multiple layers. We use the pretrained BERT_base_ where the number of transformer blocks/layers *L* is 12 and hidden size *H* is 768, while the number of self-attention heads *A* is 12. The model is fine-tuned for detecting ADRs using 5 epochs. Batch size and learning are set to 16 and 2*e* − 5, respectively.

Table 2 shows the results of the baseline models and the proposed model. It is observed that deep learning techniques in general yield better results than the conventional models, i.e., SVM and MLP. Among the conventional models, MLP performs better than SVM. We find that ADR and drug terms alone do not play a substantial role in identifying ADRs. This indicates that spotting keywords in the given sentence cannot lead to extracting adverse drug reactions effectively as the problem depends more on the context. Incorporating contextual information using word *n*-grams and semantic information using sentence embeddings improves the performance of these models. However, word *n*-grams in these models are represented as their term frequencies which are not enough for effective classification.

In deep learning models, words in the input sequence are represented as word embeddings, and hence, the contextual information is learned utilizing the semantic representation of the words in the form of embeddings through multiple layers of the network. Among deep neural networks, BERT performs better than CNN, and CNN performs better than LSTM. We find CNN performing better than LSTM because CNNs capture local patterns while LSTMs capture global patterns in the input. We observe that in most of the cases, input sequences comprise short text. Hence, information from the local key phrases which are effectively extracted by applying CNN plays a primary role in ADR extraction. LSTMs on the other hand are good at capturing long-range dependencies. When applying LSTM, the input sentence is encoded as a long example. As a result, some important phrases may not be learned as a salient feature.

We also observe the effects of different embedding models, i.e., word2vec, fasttext, and glove, on CNN and LSTM. We find that both CNN and LSTM perform better when initialized with fasttext embeddings than word2vec and glove embeddings. The fasttext model takes into account the morphology of the words by extracting information from the internal structure of the words rather than considering just the whole words in the context. Fasttext represents each word by the sum of their char *n*-grams. By considering the subword information, fasttext unlike word2vec and glove generates the embeddings for out of vocabulary words as well. The training data used for any machine learning model, no matter how big it may be, can still not include all the words in a language's vocabulary. If such unseen words are found in the test data, their representations are not generated by word2vec and glove embedding models. However, fasttext overcomes this limitation and represents the out of vocabulary words by adding the embeddings for the constituent char *n*-grams found in the vocabulary.

BERT outperforms both CNN and LSTM. The reason for the better performance of BERT is that it learns contextualized embeddings in a bidirectional way. In natural language, a word is likely to convey multiple meanings based on the context in which it is used. Word2vec, fasttext, and glove produce the same representations of a word even if it has different meanings in different contexts. BERT, on the other hand, produces context-dependent embeddings of a word. In BERT, an input word is represented by the sum of its token embeddings, sentence embeddings, and position embeddings.

The proposed model FARM-BERT outperforms all the models by yielding the *F*-scores of 89.6% and 97.6% on Twitter and PubMed datasets, respectively. FARM-BERT performs better than BERT by 2% on Twitter and by 6% on PubMed datasets. Better performance of FARM-BERT than the standard BERT indicates the effectiveness of fine-tuning BERT with FARM with the modified values of hyperparameters.

### 4.5. Comparison of Computational Performance of FARM-BERT with BERT

In this section, we compare the computational time consumed by training and testing BERT and FARM-BERT on Twitter and PubMed datasets.  Table 3 shows the computation time of training both the models for each epoch in seconds while Table 4 shows the test time of both the models in seconds. Training time of both the models on PubMed and Twitter datasets is also demonstrated in Figures 3(a) and 3(b), respectively. Similarly, the test time of both models on both datasets is demonstrated in Figure 4.

The experiments show that training BERT in each epoch takes more time than training FARM-BERT. A similar observation has been made while testing BERT and FARM-BERT. Hence, FARM-BERT works computationally faster than the standard BERT during both training and testing. FARM-BERT is computationally faster than BERT because FARM supports parallel processing. Furthermore, support for using multiple prediction heads for multitask learning also makes FARM-BERT faster than the standard BERT. The analysis of the computational performance of both of the models indicates the effectiveness of using FARM-BERT for ADR prediction instead of the standard BERT.

### 4.6. Comparison with State-of-the-Art Works

In this section, we compare the results of our proposed approach with the state-of-the-art works performed on the three datasets, i.e, PubMed dataset, Twitter dataset, and TwiMed dataset.

Table 5 tabulates the results of the proposed method and previous works performed on PubMed and Twitter datasets. *F*-scores achieved by these models are visually displayed in Figures 5(a) and 5(b), respectively.

The comparisons are made with the works performed by Cocos et al. [12], Ramamoorthy and Murugan [9], and Ding et al. [11]. The model by Cocos et al. [12] uses BLSTM which combines forward and reverse RNNs. 400-dimensional pretrained embeddings are used to initialize the embedding layer [52]. The model has been applied to the Twitter dataset. Ramamoorthy and Murugan [9] use BLSTM initialized with a combination of charCNN embedding, word2vec word embedding, and PoS embeddings. The model uses the self-attention mechanism and has been applied to the PubMed dataset. Ding et al. [11] use BGRU with a combination of charLSTM embeddings and 300-dimensional glove word representations [52] through the embedding level attention mechanism. The output of the embedding level attention layer is used as an auxiliary classifier and added to the BGRU output layer to identify ADRs. This model has been applied to both PubMed and Twitter datasets. It is evident from Table 5 that the proposed model FARM-BERT outperforms all the state-of-the-art models applied to Twitter and PubMed datasets. In terms of the *F*-score, FARM-BERT performs better than Cocos et al. [12] by approximately 14% on the Twitter dataset. It performs better than Ramamoorthy and Murugan [9] by approximately 10% on the PubMed dataset. It yields better performance than Ding et al. [11] by approximately 5% and 7% on Twitter and PubMed datasets, respectively.

Table 6 compares the results achieved by FARM-BERT with results achieved by the previous works on TwiMed corpus. *F*-scores of the models on TwiMed-Twitter and TwiMed-PubMed datasets are also demonstrated in Figures 6(a) and 6(b), respectively.

The first two models in Table 6, i.e., SVM and interactive attention network (IAN), have been used by Alimova and Solovyev [48] on the TwiMed dataset. IAN uses the attention mechanism to learn target and contextual representations. The experiments using the CNN-based method, multichannel CNN, joint AB-LSTM, and Multihop Self-Attention Mechanism (MSAM) have been performed by [47] on TwiMed corpus. The CNN-based method was proposed by Liu et al. [49] and Quan et al. [50] for relationship detection. Joint AB-LSTM was proposed by Sahu and Anand [51]. MSAM has been proposed by [29] which uses the multihop mechanism to learn complex semantic information by focusing on different segments of a sentence. It can be seen from the table that the FARM-BERT approach proposed by our work performs better than all the other approaches.

## 5. Conclusion

This work proposes BERT fine-tuned with FARM (FARM-BERT) to detect ADRs. The proposed model FARM-BERT uses parallelized preprocessing which makes it computationally faster than standard BERT and hence reasonable to use in production environments. Using multitask learning, an end-to-end solution for identifying ADRs is presented. BERT pretrained on BBC news corpus is used which is then fine-tuned with FARM to model the downstream task of detecting ADRs. Experiments are performed on Twitter, PubMed, and TwiMed datasets, and results are compared with different baseline models, i.e., SVM, MLP, CNN, LSTM, and standard BERT. Results are also compared with the other state-of-the-art works. It is shown that the proposed FARM-BERT outperforms all the baselines and state-of-the-art models yielding the *F*-scores of 89.6%, 97.6%, 84.9%, and 95.9% on Twitter, PubMed, TwiMed-Twitter, and TwiMed-PubMed datasets, respectively. Furthermore, training time and testing time taken by BERT and FARM-BERT are compared, and it is shown that FARM-BERT takes less time than BERT for both training and testing.

The results achieved by the proposed approach are quite promising; however, BERT pretrained on BBC corpus is used as the language model on the downstream task of the biomedical domain. Using a language model of a different domain does not effectively represent the linguistic details of the domain of the downstream task. Hence, the proposed approach can be further improved by pretraining the BERT language model on the biomedical text and adapting this model to the downstream task of ADR detection. We aim to address this limitation in the future by investigating the effect of pretraining BERT on the biomedical text and then fine-tuning it with FARM to detect ADRs.

## Figures and Tables

**Figure 1:** FARM-BERT architecture.

**Figure 2:** Examples of ADRs in (a) Twitter and (b) PubMed datasets.

**Figure 3:** Training time of BERT and FARM-BERT for each epoch on Twitter and PubMed datasets.

**Figure 4:** Test time of BERT and FARM-BERT on Twitter and PubMed datasets.

**Figure 5:** *F*-scores achieved by different models on Twitter and PubMed datasets.

**Figure 6:** *F*-scores yielded by different models on TwiMed dataset.

**Table 1:** Quantitative details of Twitter, PubMed, and TwiMed datasets.

Datasets	No. of documents	No. of labels	Max sentence length
Twitter	844	4	36
PubMed	6821	3	93
TwiMed-PubMed	1000	2	137
TwiMed-Twitter	625	2	64

**Table 2:** Comparison of results yielded by FARM-BERT with the results yielded by baseline models applied on Twitter and PubMed datasets.

Models	Features	Twitter			PubMed		
		*P*	*R*	*F*	*P*	*R*	*F*
SVM	Word *n*-grams	0.701	0.650	0.675	0.711	0.682	0.695
	ADR terms	0.503	0.514	0.508	0.539	0.558	0.548
	Sentence embeddings	0.604	0.644	0.624	0.671	0.611	0.641
	Word *n*-grams+ADR terms+sentence embeddings	0.729	0.688	0.708	0.717	0.706	0.711

MLP	Word *n*-grams	0.711	0.661	0.686	0.719	0.684	0.701
	ADR terms	0.512	0.524	0.518	0.521	0.544	0.532
	Sentence embeddings	0.615	0.645	0.630	0.685	0.666	0.675
	Word *n*-grams+ADR terms+sentence embeddings	0.727	0.738	0.732	0.733	0.756	0.744

LSTM	Word2vec word embeddings	0.779	0.798	0.788	0.801	0.792	0.796
	Fasttext word embeddings	0.786	0.812	0.799	0.825	0.798	0.811
	Glove word embeddings	0.771	0.782	0.776	0.810	0.786	0.798

CNN	Word2vec word embeddings	0.854	0.799	0.826	0.861	0.806	0.833
	Fasttext word embeddings	0.863	0.801	0.832	0.877	0.819	0.848
	Glove word embeddings	0..843	0.803	0.823	0.872	0.798	0.835

BERT	BERT embeddings	0.831	0.850	0.870	0.920	0.930	0.910

FARM-BERT	BERT embeddings	0.840	0.861	0.896	0.982	0.964	0.976

**Table 3:** Comparison of training time of BERT and FARM-BERT for each epoch on Twitter and PubMed datasets.

Epochs	Training time of the models			
	PubMed dataset		Twitter dataset	
	BERT	FARM-BERT	BERT	FARM-BERT
Epoch 1	604.01	360.37	192.21	152.44
Epoch 2	596.36	420.06	193.04	151.31
Epoch 3	589.01	399.42	187.22	156.51
Epoch 4	579.32	393.21	192.11	149.22
Epoch 5	574.50	391.40	192.38	153.49

**Table 4:** Comparison of test time of BERT and FARM-BERT on Twitter and PubMed datasets.

	Test time of the models	
	PubMed dataset	Twitter dataset
BERT	46.1	22.51
FARM-BERT	33.4	18.32

**Table 5:** Comparison of results yielded by FARM-BERT with the results yielded by state-of-the-art models on Twitter and PubMed datasets.

Models	Twitter			PubMed		
	*P*	*R*	*F*	*P*	*R*	*F*
Cocos et al. [12]	0.704	0.829	0.755	—	—	—
Ramamoorthy and Murugan [9]	—	—	—	0.884	0.824	0.853
Ding et al. [11]	0.785	0.914	0.844	0.867	0.948	0.906
FARM-BERT	0.84	0.861	0.896	0.982	0.964	0.976

**Table 6:** Comparison of results yielded by FARM-BERT with the results yielded by state-of-the-art models on TwiMed corpus.

Models	TwiMed-Twitter			TwiMed-PubMed		
	*P*	*R*	*F*	*P*	*R*	*F*
SVM [48]	0.752	0.810	0.778	0.799	0.681	0.728
IAN [48]	0.836	0.813	0.824	0.878	0.738	0.792
CNN-based method [49]	0.739	0.788	0.761	0.849	0.831	0.835
Multichannel CNN [50]	0.738	0.841	0.780	0.861	0.780	0.816
Joint AB-LSTM [51]	0.748	0.856	0.799	0.858	0.852	0.853
MSAM [47]	0.701	0.828	0.754	0.817	0.856	0.831
FARM-BERT	0.831	0.868	0.849	0.952	0.966	0.959

## Data Availability

The Twitter dataset on ADR data used to support the findings of this study is included within the article.
